The article "Astragalus Polysaccharides Enhance the Immune Response to OVA Antigen in BALB/c Mice" was published in 2021. Journal: Biomed Res Int.

# Astragalus Polysaccharides Enhance the Immune Response to OVA Antigen in BALB/c Mice

**DOI:** 10.1155/2021/9976079

**Published:** 2021-06-28

**Authors:** Yumei Zhou, Yuhan Zong, Zihao Liu, Haihong Zhao, Xiaoshan Zhao, Ji Wang

**Affiliations:** ^1^National Institute of TCM Constitution and Preventive Medicine, School of Chinese Medicine, Beijing University of Chinese Medicine, Beijing 100029, China; ^2^Department of Cancer Prevention, Tianjin Medical University Cancer Institute and Hospital, National Clinical Research Center for Cancer, Tianjin 300060, China

## Abstract

Vaccination has been identified as one of the most effective ways to prevent the transmission of infectious diseases in humans and animals. One of the most critical steps in vaccine development is the selection of a suitable adjuvant. Although various adjuvant candidates have been evaluated in the past few decades, only a limited amount of them are nontoxic and safe for human use. Astragalus polysaccharide (APS), due to its lack of toxicity, has been used as an immunomodulator to enhance immune responses. On the other hand, the immune effects of APS on ovalbumin are yet to be examined. Thus, in this study, we analyzed APS's effects on the immune response to ovalbumin in BALB/c mice. We have also used the classic adjuvant CpG oligodeoxynucleotide as the positive control.

## 1. Introduction

Vaccination has been established as an effective means to prevent many diseases. Improving the understanding of the mechanism of adjuvants is pivotal to harnessing the potential of existing and new adjuvants to achieve a desired immune response [1].

Traditional herb medicine as an alternative or supplemental medicine has been widely used to treat various diseases in China, Japan, and other Asian countries [2]. For example, astragalus membranaceus, which is a commonly used Chinese medicinal plant, contains polysaccharides, saponins, flavonoids, and some other components that activate the immune response and promote antibody production and immune response [3]. Astragalus polysaccharides (APS), a monomer derived from *Astragalus membranaceus*, is also one of the active components in Huangqi (Radix Astragali Mongolici), a traditional Chinese medicine that has been demonstrated in recent years to be a promising treatment for different diseases. APS has been shown to have immunomodulatory [4], antioxidant [5], antitumor [6], antidiabetes [7], and anti-inflammatory [8] activities and antiviral effects [9]. APS is nontoxic; however, its immunogenicity remains unclear.

Aluminum salts are classic adjuvants used in vaccines against hepatitis A and B, diphtheria-tetanus-pertussis (DTaP), *Haemophilus influenzae* type b (Hib), human papillomavirus (HPV), and pneumococcus infectious agents. Aluminum salts have been used safely in vaccines for more than 70 years [10]. Aluminum salts have many effects in enhancing immune effects, whereas there is a concern for the safety of aluminum adjuvants for individuals potentially predisposed to adverse neurological consequences [11]. There are many other adjuvants, such as TLR agonist adjuvants and Protollin (a complex of Proteosomes with LPS derived from Shigella flexneri). However, these adjuvants have different drawbacks, such as a lack of immunogenicity, and toxicity to the human body is a particular concern.

The article "Astragalus Polysaccharides Enhance the Immune Response to OVA Antigen in BALB/c Mice" was published in 2021. Journal: Biomed Res Int.

CpG oligonucleotides (ODN), immunomodulatory synthetic oligonucleotides designed to stimulate TLR9 (Toll-like receptor 9), are expressed on human plasmacytoid dendritic cells and B cells. CpG ODNs trigger an innate immune response characterized by the production of Th1 and proinflammatory cytokines [12]. Thus, there is a need for new, nontoxic adjuvants that are robustly immunogenic to induce both Th1 and Th2-related immune responses.

Here, we tested whether APS could enhance the immunity of vaccines. We selected OVA as an immunogen and CpG as the positive control to evaluate the effects of APS as an adjuvant for the OVA antigen in BALB/c mice.

## 2. Materials and Methods

### 2.1. Materials

Ovalbumin (Sigma), a BrdU kits (Affymetrix eBioscience), rabbit anti-mouse IgG-HRP antibody (Elabscience), and APS (Tianjin Cinorch Pharmaceutical Co., Ltd., Tianjin, China) were purchased. CpG ODN1826 (5′-TCCATGACGTTCCTGACGTT-3′) was synthesized (Sangon Biotech, Shanghai Co., Ltd.) with full chain phosphorothioate modification and PAGE-purified.

### 2.2. Histopathological Analysis by Hematoxylin and Eosin (HE) Staining

The spleen tissues were fixed in 4% paraformaldehyde and then embedded in paraffin and sliced into 4 *μ*m thick sections. The sections were then stained with hematoxylin and eosin for morphological examination using a light microscope (Olympus) at 200x magnification.

### 2.3. Animals and Immunization

Six- to eight-week-old specific pathogen-free (SPF) female BALB/c mice (Beijing Vital River Laboratory Animal Technology Co., Ltd., Beijing, China) were maintained under SPF conditions in an animal facility and given sterile water, mouse chow, and bedding. Four test groups of mice, with five per group, were immunized by intramuscular injection with 100 *μ*g of OVA, 100 *μ*g of OVA and 50 *μ*g of APS (OVA + APS), or 100 *μ*g of OVA and 50 *μ*g of CpG ODN1826 (OVA+CpG) in 200 *μ*L of sodium chloride (NaCl). The control group received 200 *μ*L NaCl.

### 2.4. Flow Cytometry of Nonspecific Spleen Cell Proliferation

Single-cell suspensions of the spleen of the mice from the four groups were prepared in a cell staining buffer (BioLegend, Inc., San Diego, CA, USA) and filtrated through a 70 *μ*m nylon mesh strainer. The viable cells were counted and suspended in the cell staining buffer at 1 × 10^7^ cells/mL; 100 *μ*L of the cell suspension was distributed into sterile Eppendorf tubes. Ten *μ*M BrdU was added to each tube for a 45-minute incubation at 37°C. After the cells were washed with the cell staining buffer, they were incubated with 1 mL of the working solution of the BrdU staining buffer at room temperature for 15 minutes and in the dark. After washing with the cell staining buffer, the cells were incubated with 100 *μ*L of DNase I at 37°C for 1 hour. Then, 5 *μ*L of anti-BrdU antibody was added to the cells to incubate for 30 minutes in the dark and at room temperature. At last, the cells were washed twice with the cell staining buffer and suspended in 0.5 mL of the same buffer for analysis by flow cytometry (FACSCalibur, BD Biosciences). In total, 10,000 events per test were collected.

The article "Astragalus Polysaccharides Enhance the Immune Response to OVA Antigen in BALB/c Mice" was published in 2021. Journal: Biomed Res Int.

### 2.5. Antigen-Specific Splenocyte Proliferation

Five mice from each group were sacrificed 8 weeks after immunization. The spleens from the same group were mixed and suspended in the RPMI-1640 medium containing 10% fetal bovine serum, 100 *μ*g/mL streptomycin, and 100 U/mL penicillin and prepared into a single-cell suspension with a cell strainer. Then, the cells were washed with phosphate-buffered saline (PBS), suspended in RPMI1640, stained with 0.4% trypan blue, and counted for the number of viable cells.

Splenocytes were added to 96-well plates at the concentration of 1 × 10^6^ cells in 200 *μ*L of RPMI1640 per well and stimulated with 8 *μ*L of ovalbumin at the final concentration of 20 *μ*g/mL or 8 *μ*L of PBS. The RPMI1640 medium was then used as the negative control. The plates were incubated in a 5% CO_2_ humidified incubator at 37°C for 72 hours. Then, 10 *μ*L of 5 mg/mL MTT was added to each well to incubate for 6 hours; 150 *μ*L of dimethyl sulfoxide was added before measurement. The extinction coefficient was measured at 570 nm. The results were expressed as the value of stimulation index (SI), calculated as SI = A570 (experimental group)/A570 (control group).

### 2.6. Enzyme-Linked Immunosorbent Assay (ELISA) Analysis for Specific IgG Antibody to OVA in Serum

The serum from the five mice in each group were collected from the immunized mice to monitor their antibody response using enzyme-linked immunosorbent assay (ELISA). Corning Costar 9018 ELISA plates (Corning Costar, Inc., Corning, NY, USA) were then coated with 2 *μ*g/mL ovalbumin overnight at 4°C. The plates were then blocked with phosphate-buffered saline with Tween 20 containing 1% bovine serum albumin (Bovogen Biologicals Pty Ltd., East Keilor, VIC, Australia). The serum were added at serial twofold dilutions. After washing, horseradish peroxidase-conjugated goat antimouse IgG (SouthernBiotech, Birmingham, AL, USA) was added. After aspirating and washing for a total of four cycles, the substrate solution (R&D system) was added to each well at 100 *μ*L/well. The plate was then incubated in the dark for 30 minutes. The reactions were stopped by adding 50 *μ*L of the stop solution to each well and read at 450 nm in 30 minutes.

The article "Astragalus Polysaccharides Enhance the Immune Response to OVA Antigen in BALB/c Mice" was published in 2021. Journal: Biomed Res Int.

### 2.7. Statistical Analysis

The cytokines in different treatment groups were compared using one-way analysis of variance followed by Tukey's multiple comparison tests of the means. The results from the BrdU analysis and SI were compared using a nonparametric Mann–Whitney *U* test (^∗^*P* < 0.05, ^∗∗∗^*P* < 0.001).

## 3. Results

### 3.1. H&E Staining of the Spleens

The size and number of the germinal centers in the OVA+APS group were significantly increased compared to those in the OVA+CpG, OVA, and NaCl groups (Figure 1).

### 3.2. Cytokine Levels in Serum

The APS-induced Th1-type cytokines, such as IFN-*γ* (average 2452 pg/mL; *P* < 0.001), are crucial in the cell-mediated response to OVA. The levels of IL-2 and IL-12 were both increased in the OVA+APS group (*P* < 0.05) compared to those in the NaCl and OVA groups. Besides, the levels of the Th2-type cytokines, such as IL-4 and IL-10, were higher than those in the NaCl and OVA groups (*P* < 0.05) (Figure 2).

### 3.3. Nonspecific Proliferation of Splenic Mononuclear Cells

The lymphocytes isolated from the mice were analyzed using the nonspecific proliferation test. The proliferation of the lymphocytes isolated from the OVA+APS immunized mice was then stimulated more significantly than other groups (Figure 3).

### 3.4. Splenocyte Stimulation Index (SI)

Upon *in vitro* restimulation with OVA, the antigen-specific proliferation of the lymphocytes isolated from the OVA and APS-immunized mice demonstrated a marked increase compared to that in the NaCl and OVA groups (Figure 4). These data suggested that the extent of proliferation was greater when the splenocytes were stimulated with OVA.

### 3.5. Serum Antibody Responses

The levels of OVA-specific IgG, IgG1, and IgG2a in the serum samples at 8 weeks after immunization were evaluated (Figures 5(a)–5(c)). As per the results, it was determined that APS- induced the highest OVA-specific IgG and IgG1 antibody responses as expected. The levels of IgG and IgG1 were higher than those in the OVA and OVA+CpG groups.

The article "Astragalus Polysaccharides Enhance the Immune Response to OVA Antigen in BALB/c Mice" was published in 2021. Journal: Biomed Res Int.

## 4. Discussion

Vaccines are designed to stimulate specific and prolonged immune responses to achieve long-term protection against infection or disease. Adjuvants, a vaccine component namely adjuvant can enhance antigen recognition by the host immune system, thereby stimulating the cellular and adaptive immune responses. Long-lasting and effective stimulation of the immune system can be achieved by conventional vaccines composed of live attenuated or inactivated pathogens. However, these vaccines are associated with several safety issues, including the mutations that may restore the pathogen's infectiousness or the incomplete inactivation of the pathogen [13]. The development of new adjuvants that are potentially efficacious as well as safe will address a significant need in modern vaccine research [14]. Although there are so many adjuvants in use, new adjuvants that are effective and nontoxic with more immune effect are needed, especially for applications for the *Brucella*, COVID-19, or other vaccines.

APS, which is extracted from *Astragalus membranaceus* roots, is generally purified by dissolution in distilled water, dialysis, and lyophilization [15]. APS has been indicated to have various biological activities, including immunomodulatory [16], anti-inflammatory [17], antioxidant, antitumor, and antiviral activities [18], among others. CpG is a kind of vaccine adjuvant that promotes Th1 immune responses and enhances the immunogenicity of many vaccines with high safety in some clinical research [19, 20]; thus, it was used as a positive adjuvant control. Ovalbumin (OVA), a 43 kDa globular protein, was used as a model vaccine antigen to evaluate the immune effect of the adjuvants.

Lymphocyte proliferation is an indicator of immune-stimulation, and it reflects the level of cellular immune response [21, 22]. Our results demonstrated that APS could induce strong cellular immune responses. As shown in Figures 3 and 4, the higher nonspecific proliferation and SI were observed in spleens in the OVA+APS group, but they were lower than that in the OVA+CpG group.

Th1 cytokines IL-2, IL-12, and IFN-*γ* are involved in facilitating the cellular immune response, and Th2 cytokines IL-4 and IL-10 mediate the humoral immune response [23, 24]. The mice immunized with OVA+APS and OVA+CpG displayed an increase in the levels of IL-2, IL-12, and IFN-*γ* compared to those in the OVA-induced mice (Figure 5). The levels of IL-4 and IL-10 in the OVA+APS group were higher than those in the OVA+CpG group (*P* > 0.05). These results indicated that APS induction could enhance both Th1- and Th2-type immune responses.

The OVA+APS and OVA+CpG treatments significantly enhanced IgG production compared to the treatment with free OVA (*P* < 0.05) (Figure 5(a)); the OVA+APS treatment induced the highest level of IgG secretion. IgG1 antibody production is a characteristic of a Th2-polarized immune response, while IgG2a antibody production is a characteristic of a Th1-polarized immune response. The ratio of IgG2a/IgG1 is indicative of a Th1-biased immune response [25, 26]. The OVA+APS treatment induced the most robust Th2-associated IgG1 responses, and OVA+CpG induced the most robust Th1-associated IgG2a responses (Figures 5(b) and 5(c)). Our study has demonstrated that APS can induce the Th1- or Th2-type immune response. Thus, APS is a potential adjuvant for the OVA-mediated immune response.

The article "Astragalus Polysaccharides Enhance the Immune Response to OVA Antigen in BALB/c Mice" was published in 2021. Journal: Biomed Res Int.

In our study, we confirmed CpG ODN1826 can induce immune response especially in vaccines which focus on Th1 type cellular immune response again. Whereas the APS adjuvant can enhance immune effect especially Th1- and Th2-type immune response, it is a new type adjuvant without toxicity. It is a new type adjuvant to be widely used in *Brucella* vaccine, COVID-19 vaccine, or other vaccines to enhance the immune effect with its effective immune effect.

Many vaccine adjuvants have been developed. Alum, MF59, and AS03 represent key benchmarks for adjuvant development; however, the tolerance to the body's immune system of many new adjuvant candidates completely differs from that of alum, inevitably increasing the safety risks [27]. The development of a new adjuvant is a long process, including the study of its mechanisms and clinical development. Understanding the mechanism of APS is critical to its potential development as an adjuvant. Here, we have conducted a preliminary study of the APS-induced immune effects. In the next study, we will explore how APS acts on the immune system and induces the immune response in the human body.

## 5. Conclusions

Astragalus polysaccharides have been shown to enhance Th1 and Th2 immune responses to OVA in BALB/c mice. APS is non-toxic and a promising candidate as a vaccine adjuvant.

## Figures and Tables

**Figure 1:** HE staining results of spleen tissues of mice in each group (×200).

**Figure 2:** Serum cytokines in each group. Note: compared with the NaCl or OVA control group, ^∗^*P* < 0.05 and ^∗∗∗^*P* < 0.001.

**Figure 3:** Nonspecific proliferation of lymphocytes in various groups. Note: compared with the NaCl or OVA control group, ^∗^*P* < 0.05 and ^∗∗∗^*P* < 0.001.

**Figure 4:** Specific proliferation in various groups. Note: compared with the NaCl or OVA control group, ^∗^*P* < 0.05 and ^∗∗∗^*P* < 0.001.

**Figure 5:** Specific IgG, IgG1, and IgG2a in serum of various groups. Note: compared with the NaCl or OVA control group, ^∗^*P* < 0.05 and ^∗∗∗^*P* < 0.001.

The article "Astragalus Polysaccharides Enhance the Immune Response to OVA Antigen in BALB/c Mice" was published in 2021. Journal: Biomed Res Int.

## Data Availability

All data are available in this paper.
